The article "SrFexNi1−xO3−δ Perovskites Coated on Ti Anodes and Their Electrocatalytic Properties for Cleaning Nitrogenous Wastewater" was retracted in 2023. Reasons: original data or images not available; unreliable results or conclusions; concerns about the data.

# SrFe*_x_*Ni_1−*x*_O_3−δ_ Perovskites Coated on Ti Anodes and Their Electrocatalytic Properties for Cleaning Nitrogenous Wastewater

**DOI:** 10.3390/ma12030511

**Published:** 2019-02-08

**Authors:** Yuqing Zhang, Zilu Jin, Lijun Chen, Jiaqi Wang

**Affiliations:** School of Chemical Engineering and Technology, Tianjin University, Tianjin 300350, China; a1090699180@tju.edu.cn (Z.J.); lijunchen@tju.edu.cn (L.C.); wangjiaqi1011@tju.edu.cn (J.W.)

**Keywords:** ferrum doping, SrNiO_3_, perovskite, electrocatalysis, nitrogenous wastewater

## Abstract

Perovskites (ABO_3_), regarded as the antioxidative anode materials in electrocatalysis to clean nitrogenous wastewater, show limited oxygen vacancies and conductivity due to their traditional semiconductor characteristic. To further improve the conductivity and electrocatalytic activity, the ferrum (Fe) element was first doped into the SrNiO_3_ to fabricate the SrFe*_x_*Ni_1−*x*_O_3−δ_ perovskites, and their optimum fabrication conditions were determined. SrFe*_x_*Ni_1−*x*_O_3−δ_ perovskites were coated on a titanium (Ti) plate to prepare the SrFe*_x_*Ni_1−*x*_O_3−δ_/Ti electrodes. Afterward, one SrFe*_x_*Ni_1−*x*_O_3−δ_/Ti anode and two stainless steel cathodes were combined to assemble the electrocatalytic reactor (ECR) for cleaning simulated nitrogenous wastewater ((NH_4_)_2_SO_4_ solution, initial total nitrogen (TN) concentration of 150 mg L^−1^). Additionally, SrFe*_x_*Ni_1−*x*_O_3−δ_ materials were characterized using Fourier Transform Infrared (FT-IR), Raman spectra, X-Ray Diffraction (XRD), Energy Dispersive X-ray (EDX), Electrochemical Impedance Spectroscopy (EIS) and Tafel curves, respectively. The results indicate that SrFe*_x_*Ni_1−*x*_O_3−δ_ materials are featured with the perovskite crystal structure and Fe is appreciably doped into SrNiO_3_. Moreover, the optimum conditions for fabricating SrFe*_x_*Ni_1−*x*_O_3−δ_ were the reaction time of 120 min for citrate sol-gel, a calcination temperature of 700 °C, and Fe doping content of *x* = 0.3. SrFe_0.3_Ni_0.7_O_2.85_, and perovskite performs attractive electrocatalytic activity (TN removal ratio of 91.33%) and ECR conductivity of 3.62 mS cm^−1^ under an electrocatalytic time of 150 min. Therefore, SrFe*_x_*Ni_1−*x*_O_3−δ_ perovskites are desirable for cleaning nitrogenous wastewater in electrocatalysis.

## 1. Introduction

With rapid industrialization development, nitrogenous wastewater massively generated by the chemical industry, municipal engineering, and agricultural life leads to a serious threat to humankind and the ecosystem [1]. Various treatment technologies have been developed to remove the nitrogenous contaminations in wastewater, such as ion exchange [2], the biochemical method [3], breakpoint chlorination [4], and adsorption [5]. However, these treatments have some disadvantages (moderate environment, the introduction of additional chemicals in water and secondary pollution, etc.), limiting their application [6]. Electrocatalysis with the metal oxides anode has attracted widespread concerns in cleaning nitrogenous wastewater owing to its high efficiency, clean oxidation, and easy controllability [7,8]. For example, Okanishi et al. [9] used the SnO_2_-modified Pt electrocatalyst to oxidize the ammonia and its activation energy realized 58 kJ mol^−1^. Reyter et al. [10] removed the nitrate using the electrochemical method with the Ti/IrO_2_ anode and NH_3_ conversion reached 82% at a current density of 80 mA cm^−2^. Nevertheless, the traditional coated anode relies on the noble or rare metal oxides (IrO_2_, Ta_2_O_5_, RuO_2_, et al.) [11].

Perovskites, as bimetallic oxides (ABO_3_), can be used as the anodic coating in electrocatalytic processes due to their low cost, abundance, and easy modification [12,13]. In the band structure of perovskite, the conduction band is determined by the 3d orbit of the B-site element [14]. The increase of 3d electrons in the B-site element enhances the electrocatalytic activity of perovskite by virtue of more electrons remaining in an excited state (valence band). Consequently, the choice of the B-site element is extremely crucial, which destines the band structure and electrocatalytic activity of perovskite [15]. The whole system of perovskite keeps electroneutrality and satisfies the restriction of tolerance factor (*t*) shown in Equation (1).

(1) $$t=\frac{R_{A}+R_{O}}{\sqrt{2}(R_{O}+R_{B})}$$

where *R*_A_, *R*_B_, and *R*_O_ stand for the radiuses of A-site cation, B-site cation, and oxygen anion (O^2−^) in the cubic perovskite structure, which can be only formed when *R*_A_ ≥ 90 pm, *R*_B_ ≥ 51 pm, and 0.75 ≤ *t* ≤ 1.0 [16,17]. Meanwhile, the more closely *t* approaches 1.0, the more stable the perovskite structure is. Accordingly, the proper A-site element stabilizes the electron structure and crystal form of perovskite. Mori et al. [18] synthesized an epitaxial La_0.8_Sr_0.2_CoO_3_ perovskite for the cathode, and its calculated *t* was equal to 0.8655.

Nickel (Ni) has the outermost electron configuration of 3d^8^4s^2^ with the abundant 3d electrons and empty 3d orbits among the transition metal elements (Mn: 3d^5^4s^2^, Fe: 3d^6^4s^2^, Co: 3d^7^4s^2^ and Cu: 3d^10^4s^1^) in the fourth period. Therefore, when Ni stands for the B-site element of ABO_3_, perovskite is expected to possess excellent electrocatalytic activity and appropriate conductivity. Moreover, in nickel-based perovskite of ABO_3_ (B = Ni), the strontium (Sr) element in the A-site can more strongly stabilize the cubic crystal construction of perovskite (*t* = 0.9704) compared with LaNiO_3_ (*t* = 0.9140), CaNiO_3_ (*t* = 0.9027) and BaNiO_3_ (*t* = 1.034) [19]. Oxygen vacancies in perovskite can provide more active sites and hydroxyl radicals (·OH) for electrocatalysis, significantly contributing to electron transfer during the reaction. In order to form more oxygen vacancies in SrNiO_3_ perovskite and then enhance its electrocatalytic properties, ferrum (Fe) can be doped and partially substitute the Ni element in the B-site, because they have similar electronegativity (Fe: 1.8, Ni: 1.8) and atomic radii (Fe: 124.1 pm, Ni: 124.6 pm). Moreover, Fe (III) and Ni (IV) show different valence states in favor of delivering electrons and forming oxygen vacancies according to the electroneutrality principle [20]. Therefore, based on the above analysis, SrFe*_x_*Ni_1−*x*_O_3−δ_ perovskites through doping Fe element into the SrNiO_3_ perform the better conductivity and electrocatalytic activity.

NH_4_^+^ represents a common contaminant in nitrogenous wastewater and the widely accepted mechanism for removing NH_4_^+^ in wastewater is the electrochemical oxidation during the electrocatalysis [21]. The ·OH can efficiently oxidize the NH_4_^+^ into N_2_ on the anode. Zhou et al. [22] degraded the ammonia nitrogen (NH_4_^+^-N) in wastewater by reverse electrodialysis (RED), and NH_4_^+^-N removal ratio reached 25% with the initial NH_4_^+^-N concentration of 10 mg L^−1^. Vlyssides et al. [23] treated the domestic wastewater (NH_4_^+^-N concentration of 150 mg L^−1^, pH = 6) through electrocatalysis and NH_4_^+^-N was reduced by 43.3% at the residence time of 30 min. In summary, the electrocatalytic method is expected to clean the wastewater containing NH_4_^+^.

In this paper, to improve the conductivity and electrocatalytic activity for removing NH_4_^+^ during the electrocatalysis, low-cost SrFe*_x_*Ni_1−*x*_O_3−δ_ perovskites were fabricated by doping Fe into SrNiO_3_, and their optimum fabrication conditions were determined. Moreover, SrFe*_x_*Ni_1−*x*_O_3−δ_ perovskites were coated on the Ti plate to prepare the SrFe*_x_*Ni_1−*x*_O_3−δ_/Ti electrodes and the electrocatalytic reactor (ECR) was assembled with the SrFe*_x_*Ni_1−*x*_O_3−δ_/Ti anode to clean simulated nitrogenous wastewater. Perovskite-type SrFe*_x_*Ni_1−*x*_O_3−δ_ structure was testified and Fe was evidently doped into the SrNiO_3_ matrix. Herein, SrFe*_x_*Ni_1−*x*_O_3−δ_ perovskites achieve attractive total nitrogen (TN) removal ratio and conductivity, indicating that they are suitable to clean nitrogenous wastewater in electrocatalysis.

## 2. Experimental

### 2.1. Materials and Reagents

*N*,*N*-dimethylacetamide (DMAc, AR grade, 99.5%), acetylene black (AR grade, 99.0%) and potassium bromide (KBr, AR grade, 99.0%) were provided by Tianjin Kemiou Chemical Reagent Co., Ltd. (Tianjin, China). Polyvinylidene fluoride (PVDF, 1015) was purchased from Solvay Co., Ltd. (Shanghai, China). Ammonium sulphate ((NH_4_)_2_SO_4_, AR grade, 99.0%), ferric nitrate (Fe(NO_3_)_3_·9H_2_O, AR grade, 99.5%), strontium nitrate (Sr(NO_3_)_2_, AR grade, 99.5%), nickel nitrate (Ni(NO_3_)_3_·6H_2_O, AR grade, 98.0%) and potassium persulfate (K_2_S_2_O_8_, AR grade, 99.5%) were supplied by Tianjin Yuanli Chemical Engineering Co., Ltd. (Tianjin, China). Sodium hydroxide (NaOH, AR grade, 99.0%) was obtained from Tianjin Guangfu Technology Development Co., Ltd. (Tianjin, China). Citric acid (C_6_H_8_O_7_·H_2_O, AR grade, 99.5%) was brought from Tianjin North Tianyi Chemicals Co., Ltd. (Tianjin, China). All reagents and chemicals were used as received.

### 2.2. Fabrication of the SrFe_x_Ni_1−x_O_3−δ_ Perovskites

SrFe*_x_*Ni_1−*x*_O_3−δ_ perovskites are fabricated using the citrate sol-gel method, which could be clearly observed from Figure 1 [24,25]. Firstly, stoichiometric amount of corresponding metal raw materials was determined, and the molar ratio of Sr: Ni: Fe: citric acid = 1: 1−*x*: *x*: 2.5, where *x* represented the doping content of Fe (*x* = 0, 0.1, 0.2, 0.3, 0.4 and 0.5). Then metal nitrates were fully dissolved in moderate deionized water to derive metallic ions aqueous solution. The mixture of both metallic ions, aqueous solution, and citric acid gently reacted at 80 °C for an appropriate time to form citrate complexation under magnetic stirring (rotational speed of 120 rpm), then dried (120 °C, 12 h) to evaporate the excess water in citrate sol-gel. Finally, precursors of SrFe*_x_*Ni_1−*x*_O_3−δ_ were calcined in a muffle furnace through a temperature-programmed route, which was linearly heated to 300 °C and maintained for 1 h, then kept at high temperature (600–750 °C) for 2 h under an air atmosphere (heating rate of 5 °C min^−1^). The desired SrFe*_x_*Ni_1−*x*_O_3−δ_ (*x* = 0, 0.1, 0.2, 0.3, 0.4 and 0.5) perovskites were obtained. In this work, the effect of reaction time for citrate sol-gel, calcination temperature, and doping content of Fe were discussed for fabricating SrFe*_x_*Ni_1−*x*_O_3−δ_ perovskites. 

### 2.3. Preparation of the SrFe_x_Ni_1−x_O_3−δ_/Ti Anode

Preparation of the SrFe*_x_*Ni_1−*x*_O_3−δ_/Ti anode is schematically displayed in Figure 2. Firstly, a titanium (Ti) plate (Grade TA2, 80.0 mm × 17.0 mm × 1.8 mm) was polished to remove the superficial oxide layer, degreased in hot detergent, and then etched by sharp blades to produce a rough grid surface, which served as the Ti substrate [26]. Afterward, anodic materials mentioned in Table 1 (SrFe*_x_*Ni_1−*x*_O_3−δ_ perovskites, acetylene black, PVDF and DMAc in a mass ratio of 56:7:7:30) [27] were fully mixed into a viscous paste and uniformly coated on the Ti substrate with a spatula. Finally, the SrFe*_x_*Ni_1−*x*_O_3−δ_/Ti anode was prepared after being dried at 80 °C for 2 h.

### 2.4. Assembly of Electrocatalytic Reactor (ECR)

As shown in Figure 3, the ECR was a single compartment reactor (height of 120.0 mm, bottom diameter of 93.0 mm) and constructed with one anode and two cathodes: SrFe*_x_*Ni_1−*x*_O_3−δ_/Ti as the anode and stainless steels as the cathodes. All the electrodes were vertically fixed with a constant gap (20.0 mm) and both sides of Ti substrate (effective area of 5.10 cm^2^) were coated with the electrode materials. Simulated nitrogenous wastewater ((NH_4_)_2_SO_4_ solution, volume of 300 mL, initial TN concentration of 150 mg L^−1^) was intermittently poured into the ECR and forced to flow in turbulence by a magnetic stirrer (rotational speed of 120 rpm). ECR was powered just by a source of direct current (DC) connecting the amperemeter and slide rheostat with copper wires. Electrocatalytic current could be directly monitored from the amperemeter and the electrocatalytic current density was calculated by Equation (2). In addition, the electrocatalytic voltage was read by the digital multimeter between anode and cathode. The resistance, conductivity, and power density of ECR could be derived from Equations (3)–(5), respectively.

(2) $$i=\frac{I}{S}$$

(3) $$r=\frac{U}{I}$$

(4) $$\kappa =\frac{L}{r\times S}$$

(5) P=U×i

where *I* is the electrocatalytic current (A), *U* is the electrocatalytic voltage (V), *S* is the effective surface area of anode (cm^2^), *L* is the gap between anode and cathode (cm), *r* is the resistance of ECR (Ω), κ is the conductivity of ECR (mS cm^−1^), *P* is the electrocatalytic power density of ECR (mW cm^−2^), and *i* is the electrocatalytic current density of anode (mA cm^−2^). Current density mentioned in this paper referred to the electrocatalytic current density of anode and all the experimental results were measured at 25 ± 2 °C.

### 2.5. Measurement of Total Nitrogen (TN) Concentration

(NH_4_)_2_SO_4_ solution was selected as the simulated nitrogenous wastewater in various TN concentrations [28]. According to the discharge standard of pollutants for municipal wastewater treatment plant in China (GB 18918-2002, Class I-A Standard [29]), the TN concentrations before and after treatment by ECR were set as 150 mg/L and ≤ 15 mg/L, respectively. The TN concentration was determined by the alkaline potassium persulphate digestion UV spectrophotometric method (HJ 636-2012 [30]), whose details were provided in the Supplementary Information (Figure S1 and Table S1). The TN removal ratio was calculated by Equation (6):

(6) $$R=\frac{C_{0}-C}{C_{0}}\times 100\%$$

where *R* is the TN removal ratio (%), *C*_0_ and *C* are the TN concentrations (mg L^−1^) of the nitrogenous wastewater before and after treatment, respectively.

### 2.6. Characterizations and Analysis Methods

#### 2.6.1. Scanning Electron Microscope (SEM) and Energy Dispersive X-ray (EDX) Studies

Samples were sputtered with gold and their superficial morphologies were observed under the S4800 SEM (Hitachi, Tokyo, Japan) with a resolution of 1 nm. In addition, the relative content of elements in SrFe*_x_*Ni_1−*x*_O_3−δ_ was analyzed by EDX system coupled with the SEM.

#### 2.6.2. Fourier Transform Infrared (FT-IR) Studies

SrFe*_x_*Ni_1−*x*_O_3−δ_ perovskite powders of 1 mg were dried, pressed into the pellets with KBr of 100 mg, and then preserved under vacuum. The FT-IR spectra of SrFe*_x_*Ni_1−*x*_O_3−δ_ perovskite pellets were collected on an Avatar 370 spectrometer (Thermo Nicolet Corp., Billerica, GA, USA) with a wavelength coverage of 400–4000 cm^−1^ and a resolution of 0.1 cm^−1^.

#### 2.6.3. Raman Analysis

The Raman spectra of SrFe*_x_*Ni_1−*x*_O_3−δ_ materials were recorded using a high-resolution HR800 Raman spectrometer (Horiba, Montpellier, France) with a 532 nm laser beam as a light source. The laser was incident on the samples in a 2 μm diameter spot through a standard ×50 microscope objective lens and the accumulation time was 60 s for spectral measurement. The baseline of the Raman spectra was corrected with a silicon wafer.

#### 2.6.4. X-Ray Diffraction (XRD) Studies

All the SrFe*_x_*Ni_1−*x*_O_3−δ_ samples were tested on a Bruker D8 Advance diffractometer (Bruker, Karlsruhe, Germany) using Cu Kα (λ = 0.154184 nm) radiation source filtered by a Ni thin plate. The XRD data were collected over the range of 2θ = 10–80°.

#### 2.6.5. Electrochemical Studies

Electrochemical studies were carried out in the Reference 3000 electrochemical workstation (Gamry, Warminster, America) equipped with a three-electrode system. SrFe*_x_*Ni_1−*x*_O_3−δ_ materials of 1.8 mg were dispersed with ethanol of 2 mL and 0.5% Nafion of 0.05 mL under ultrasound, then the mixtures were dropped on the rotating disk electrode (RDE710, electrode area of 0.19625 cm^2^, rotating speed of 1000 rpm), which were dried and served as the working electrodes. The reference electrode and counter electrode were the saturated calomel electrode (SCE) and platinum wire, respectively. Electrochemical tests, including Electrochemical Impedance Spectroscopy (EIS) and Tafel curve, were studied in Na_2_SO_4_ (0.5 mol L^−1^) electrolyte solution under air atmosphere. The Tafel curve was performed with the sweep rate of 10 mV s^−1^ in a potential range from open potential to 0.6 V. EIS was performed with an amplitude of 5 mV from 100 kHz to 0.01 Hz. The relationship between current density and overpotential satisfies Equation (7), which can be applied and deduced into the low range of overpotential to calculate the value of exchange current density.

(7) η=a+b×logi

where *η* was the overpotential (mV) and *i* was the current density. When *η* = 0, the exchange current density (*i*_0_) could be deduced.

## 3. Results and Discussion

### 3.1. Optimum Fabrication Conditions of SrFe_x_Ni_1−x_O_3−δ_ Materials

The appropriate conditions of ECR, namely the SrFe*_x_*Ni_1−*x*_O_3−δ_ perovskites amount of 0.09804 g cm^−2^ coated on the anode, current density of 11.76 mA cm^−2^ and electrocatalytic time of 30 min, are determined in the Supplementary Information (Figures S2 and S3). Based on the above conditions of ECR, optimum fabrication conditions of SrFe*_x_*Ni_1−*x*_O_3−δ_ perovskites (reaction time for citrate sol-gel, calcination temperature and doping content of Fe in SrFe*_x_*Ni_1−*x*_O_3−δ_) need to be further confirmed and their electrocatalytic properties are studied in cleaning the nitrogenous wastewater. Moreover, the chemical formulas and oxygen vacancy values (δ) of SrFe*_x_*Ni_1−*x*_O_3−δ_ perovskites with different doping content values (*x*) can be determined by the electroneutrality.

#### 3.1.1. Effect of Reaction Time for Citrate Sol-Gel on Electrocatalytic Properties of SrFe*_x_*Ni_1−*x*_O_3−δ_

During the fabrication of SrFe*_x_*Ni_1−*x*_O_3−δ_ perovskites (calcination temperature of 700 °C), the effect of reaction time for citrate sol-gel on the electrocatalytic properties (TN removal ratio and conductivity of ECR) is illustrated in Figure 4. Obviously, TN removal ratio and the conductivity of ECR improve along with the reaction time for citrate sol-gel from 30–120 min, and then basically remain unchanged over 120 min. The results suggest the complexation between citric acid and metallic ions (Sr^2+^, Ni^3+^, and Fe^3+^) gradually increases in the citrate sol-gel, which is beneficial to fabricate the SrFe*_x_*Ni_1−*x*_O_3−δ_ perovskites and promote their electrocatalytic properties within 120 min. Moreover, among the SrFe*_x_*Ni_1−*x*_O_3−δ_ (*x* = 0, 0.1, 0.2, 0.3, 0.4 and 0.5) materials, SrFe_0.3_Ni_0.7_O_2.85_ achieves the superior TN removal ratio (56.20%) and conductivity of ECR (3.62 mS cm^−1^) at the reaction time of 120 min for citrate sol-gel. Thus, the optimum reaction time for citrate sol-gel is chosen as 120 min, over which the conductivity of ECR and the TN removal ratio have no obvious improvements.

#### 3.1.2. The Effect of Calcination Temperature on the Electrocatalytic Properties of SrFe*_x_*Ni_1−*x*_O_3−δ_

In light of the reaction time of 120 min for the citrate sol-gel, the effect of calcination temperature on the electrocatalytic properties of SrFe*_x_*Ni_1−*x*_O_3−δ_ clearly presents in Figure 5. With improving the calcination temperature for SrFe*_x_*Ni_1−*x*_O_3−δ_, both the conductivity of ECR and the TN removal ratio firstly increase and then drop, of which the peak values appear at 700 °C. This is because the SrFe*_x_*Ni_1−*x*_O_3−δ_ materials gradually form and stabilize the perovskite-type structure when their calcination temperatures increase from 600–700 °C. However, in terms of SrFe*_x_*Ni_1−*x*_O_3−δ_ materials, higher calcination temperatures (750 °C) probably destroy their crystal structure and framework [31]. Similarly, among the SrFe*_x_*Ni_1−*x*_O_3−δ_ (*x* = 0, 0.1, 0.2, 0.3, 0.4 and 0.5) materials, SrFe_0.3_Ni_0.7_O_2.85_ achieves superior electrocatalytic activity (TN removal ratio of 56.20%) and ECR conductivity of 3.62 mS cm^−1^ at the calcination temperature of 700 °C. Thereby, the optimum calcination temperature for fabricating SrFe*_x_*Ni_1−*x*_O_3−δ_ materials is considered as 700 °C.

#### 3.1.3. The Effect of the Doping Content of Fe in SrFe*_x_*Ni_1−*x*_O_3−δ_ on Electrocatalytic Properties

With regard to the optimum fabrication conditions (reaction time of 120 min for citrate sol-gel and a calcination temperature of 700 °C), the SrFe*_x_*Ni_1−*x*_O_3−δ_ materials with different doping contents of Fe (*x* value) were coated on the anode in ECR, and their electrocatalytic properties were recorded in Table 2. The electrocatalytic voltage and power density of ECR with SrFe*_x_*Ni_1−*x*_O_3−δ_/Ti anode firstly drop and then ascend, raising the *x*. Additionally, both the TN removal ratio and conductivity of ECR give the inverse tendency plotted in Figure 6 that results from the increase of oxygen vacancies and the decline of *t* with the increase of *x* in SrFe*_x_*Ni_1−*x*_O_3−δ_ perovskites. Among the SrFe*_x_*Ni_1−*x*_O_3−δ_ (*x* = 0, 0.1, 0.2, 0.3, 0.4 and 0.5) materials, SrFe_0.3_Ni_0.7_O_2.85_ has the highest conductivity of ECR (3.62 mS cm^−1^) and TN removal ratio (56.20%), manifesting its superior conductivity and electrochemical activity. Therefore, the optimum doping content of Fe in SrFe*_x_*Ni_1−*x*_O_3−δ_ is *x* = 0.3.

In the SrFe*_x_*Ni_1−*x*_O_3−δ_ perovskites, electron exchange process of B-site elements takes place due to different ionic valence states between Fe (III) and Ni (IV), promoting the electronic and conductivity and the electron transmission capacity. Meanwhile, the Fe element has more empty 3d orbits (Fe: 3d^6^4s^2^, four empty 3d orbits) and can be beneficial to deliver the electrons as compared with the Ni element (Ni: 3d^8^4s^2^, two empty 3d orbits) in the B-site. With raising the *x*, low-valent substitution in the B-site increases the oxygen vacancies according to the electroneutrality, which can also improve the ionic conductivity and electrocatalytic reactivity of SrFe*_x_*Ni_1−*x*_O_3−δ_ perovskites. However, the large *x* value relates to the low *t* value, which consequently leads to the oxygen octahedral distortion of perovskite owing to the Jahn-Teller effect, and the deviation from the standard cubic crystal structure conversely decreases the electrocatalytic reactivity and conductivity by doping [32,33].

The relationship of the *x* value in SrFe*_x_*Ni_1−*x*_O_3−δ_ perovskite materials and their characteristic parameters (oxygen vacancy value (δ), tolerance factor (*t*), and 3d electron number in the B-site) is clearly shown in Figure 7. The increasing *x* value in SrFe*_x_*Ni_1−*x*_O_3−δ_ naturally raises the oxygen vacancy value (δ) in accordance with the electroneutrality principle, which significantly avails to provide more electrocatalytic active sites and oxidative ·OH, as well as to enhance the conductivity in the perovskite. Oppositely, both the *t* value and 3d electron number in the B-site decreases with the *x* value in SrFe*_x_*Ni_1−*x*_O_3−δ_ perovskite materials, limiting their electrocatalytic activity and conductivity. The *t* values of SrFe*_x_*Ni_1−*x*_O_3−δ_ materials are totally over 0.92 (*t* = 0.9704–0.9296) and in the range of tolerance factor restriction (0.75 ≤ *t* ≤ 1.0), agreeing with the characteristic of the perovskite structure. From the results and analysis, the optimum *x* value in SrFe*_x_*Ni_1−*x*_O_3−δ_ perovskites (*x* = 0.3) reveals the balance among oxygen vacancy, 3d electron number in the B-site, and the tolerance factor of the perovskite.

### 3.2. The Effect of Electrocatalytic Time on TN Concentration

In order to investigate the effect of electrocatalytic time and further decrease the TN concentration of wastewater to a lower level, ECR with the SrFe_0.3_Ni_0.7_O_2.85_/Ti anode (current density of 11.76 mA cm^−2^ and SrFe*_x_*Ni_1−*x*_O_3−δ_ materials amount of 0.09804 g cm^−2^) is applied to treat the nitrogenous wastewater under the optimum conditions for fabricating SrFe*_x_*Ni_1−*x*_O_3−δ_ materials (reaction time of 120 min for citrate sol-gel and calcination temperature of 700 °C). TN concentrations are measured at the corresponding electrocatalytic time, and their variation trend is shown in Figure 8. With the increase of electrocatalytic time, TN concentration of wastewater in ECR gradually declines and reaches below 15 mg L^−1^ at an electrocatalytic time of 150 min. At the same time, wastewater treated by ECR satisfies the discharge standard of pollutants for municipal wastewater treatment plants in China (GB 18918-2002 [29], Class I-A Standard, TN ≤ 15 mg L^−1^) with a TN removal ratio of 91.33% (from 150 mg L^−1^ to 14.62 mg L^−1^). In the range of low TN concentrations (15–60 mg L^−1^), the variation trend of the TN concentration with the electrocatalytic time is evidently slow, possibly contributing from the reduction of the concentration driving force for limiting the electrocatalytic efficiency. On the aspect of the wastewater quality standard, the appropriate electrocatalytic time can be chosen as 150 min, over which the nitrogenous wastewater treated by ECR meets the discharge standard of pollutants for municipal wastewater treatment plants in China (GB 18918-2002 [29], Class I-A Standard, TN ≤ 15 mg L^−1^). In conclusion, the optimum operating conditions and performance of ECR with SrFe*_x_*Ni_1−*x*_O_3−δ_/Ti anode are summarized in Table 3.

### 3.3. Characterization of SrFe_x_Ni_1−x_O_3−δ_

SrFe*_x_*Ni_1−*x*_O_3−δ_ (*x* = 0, 0.1, 0.2, 0.3, 0.4 and 0.5) materials were fabricated under the optimum conditions (reaction time of 120 min for citrate sol-gel and calcination temperature of 700 °C). Then the corresponding SrFe*_x_*Ni_1−*x*_O_3−δ_ materials were characterized as described below.

#### 3.3.1. SEM Studies of SrFe_x_Ni_1−x_O_3−δ_ and SrFe_x_Ni_1−x_O_3−δ_/Ti Anodes

According to the optimum doping content of Fe (*x* = 0.3) for SrFe*_x_*Ni_1−*x*_O_3−δ_ materials, SrFe_0.3_Ni_0.7_O_2.85_ has decent electrocatalytic properties. Furthermore, SrFe_0.3_Ni_0.7_O_2.85_ material and the anodic materials of the SrFe_0.3_Ni_0.7_O_2.85_/Ti anode are characterized through SEM and their surface morphologies are shown at different magnifications (Figure 9). SrFe_0.3_Ni_0.7_O_2.85_ material exhibits the blocky solid-solution shape (particle size of 10–100 μm) in Figure 9a,b, triggered by high calcination temperature and lasting calcination time during the fabrication process. In addition, the clear cracks of SrFe_0.3_Ni_0.7_O_2.85_ material can be also observed from Figure 9a. Moreover, Figure 9c,d show the adhesive phenomena and roughness on the coated surface of SrFe_0.3_Ni_0.7_O_2.85_/Ti anode, of which the loose morphology facilitates the mass transfer and the contact between contaminants and electrode surface.

#### 3.3.2. FT-IR and Raman Analysis of SrFe*_x_*Ni_1−_*_x_*O_3−δ_

FT-IR spectra of perovskite-type SrNiO_3_ and SrNiO_3_ precursor were displayed in Figure 10. The SrNiO_3_ precursor was fabricated without the heat treatment and calcination process and the SrNiO_3_ perovskite was subsequently fabricated after heating and calcining the SrNiO_3_ precursor. In accordance with the literature [34,35], the wide and intensive absorption peak approximately ranging from 3000–3500 cm^−1^ can be assigned to the stretching vibration of O–H. Characteristic adsorption peaks at 640 cm^−1^, 895 cm^−1^, and 1074 cm^−1^ represent the C–H vibration. Meanwhile, the peaks of 1388 cm^−1^ and 1589 cm^−1^ belong to the stretching vibration of COO^−^, mainly contributing from the residual citric acid in the SrNiO_3_ precursor. Furthermore, the out-plane vibration of 812 cm^−1^ can be ascribed to nitrate radicals in the raw reagent.

As shown in Figure 11a, all the SrFe*_x_*Ni_1−*x*_O_3−δ_ materials basically perform the same tendency in the FT-IR spectra. The low-frequency adsorption of 570 cm^−1^ possibly results from translational motion between the A-site cation and BO_6_ octahedron, suggesting the ionic vibration environment of the A-site element [36]. The intensive absorption band appearing at 735 cm^−1^ can be ascribed to the A-O-B stretching vibration and it is slightly split into two peaks in Fe-doped SrNiO_3_ due to the B-site difference of the ionic radius and the valence state [37]. The well-resolved peak of 858 cm^−1^ is considered to belong to the B–O stretching in perovskite compounds [38]. In addition, the vibrational peaks at the high-frequency region can be assigned to the asymmetric stretch (1450 cm^−1^, 2482 cm^−1^) and bend (1068 cm^−1^, 1770 cm^−1^) of the BO_6_ octahedra [39]. The absorption peak of Fe_2_O_3_ is not detected in the FT-IR spectroscopy, indicating that Fe element does center into the lattice of SrNiO_3_ perovskite. Moreover, the doping of the Fe element has not changed the perovskite framework structure, and its doping content (*x*) in SrFe*_x_*Ni_1−*x*_O_3−δ_ can reach *x* = 0.5.

The Raman spectra of SrFe*_x_*Ni_1−*x*_O_3−δ_ are exhibited in Figure 11b. The Raman active mode located around 143 cm^−1^ is associated with the vibration of the oxygen ion and A-site cation, reflecting the Raman information of Sr–O [40]. The mode appearing at 174 cm^−1^ is related to the bending vibration of oxygen and B-site cation, proving the occurrence of O–Ni–O and O–Fe–O in perovskite [41]. The Raman peak at 489 cm^−1^ is assigned to the breathing vibration of oxygen in (Ni/Fe)O_6_ octahedra, which is sensitive to the B-site substitution [42]. The Raman spectra can clearly identify the effect of B- and the A-site cations, which contributes to the perovskite structure of ABO_3_.

#### 3.3.3. XRD Analysis of SrFe*_x_*Ni_1−_*_x_*O_3−δ_

Further refined characterization of SrFe*_x_*Ni_1−*x*_O_3−δ_ materials is conducted by XRD analysis in Figure 12. All the XRD diffraction peaks emerging at 29.6°, 32.8°, 37.3°, 44.1°, 43.4°, and 62.9° are sharp and intensive, certifying the brilliant crystallinity of SrFe*_x_*Ni_1−*x*_O_3−δ_ materials. Above all, XRD patterns are featured with pure perovskite-type SrNiO_3_ (PDF#28-1242) and the doping of Fe element does not change the single perovskite phase [43,44], which agrees with the FT-IR and Raman analysis. No diffraction peaks of Fe_2_O_3_, Fe_3_O_4_, NiO, SrO or other impurities can be observed in the XRD patterns, demonstrating that Fe element is successfully doped into the crystal lattice of perovskite-type structure [45]. According to the results of analysis software (Jade 6.5), the average crystallite sizes are in the range of 432–485 nm for the SrFe*_x_*Ni_1−*x*_O_3−δ_ materials. Moreover, the FWHM (full width at half maximum) value for the XRD patterns of SrFe*_x_*Ni_1−*x*_O_3−δ_ materials is calculated as 0.332 at the sharpest XRD peak (2θ = 32.8°), which is located in the range (0.1–0.5) of the common crystal material (α-quartz, mica, corundum, diamond, et al.).

#### 3.3.4. EDX Analysis of SrFe*_x_*Ni_1−_*_x_*O_3−δ_

Figure 13 shows the EDX spectrum of SrFe_0.3_Ni_0.7_O_2.85_ perovskite, in which the Sr, Ni, Fe, and O elements exist, confirming that the Fe element is present in the doped SrNiO_3_ perovskite. The C element and other impurity elements are not also found through the EDX analysis, suggesting that the citric acid is obviously decomposed during the heating and calcination process for fabricating the SrFe_0.3_Ni_0.7_O_2.85_ perovskite. Moreover, the relative content of elements in SrFe_0.3_Ni_0.7_O_2.85_ perovskite can be obtained in Table 4 and the molar ratio of Sr, Ni, Fe, and O elements in the tested material is about 1.00: 0.73: 0.34: 2.58, which is close to the theoretical molar ratio of SrFe_0.3_Ni_0.7_O_2.85_ perovskite.

#### 3.3.5. Electrochemical Impedance Spectroscopy (EIS) and Tafel Curves Analysis of SrFe*_x_*Ni_1−_*_x_*O_3−δ_

The electrochemical results (EIS and Tafel curves) of SrFe*_x_*Ni_1−*x*_O_3−δ_ perovskites present in Figure 14 and their electrochemical parameters (*R*_ct_ and *i*_0_) are obtained in Table 5. As can be seen in Figure 14a, the high frequency-region of EIS presents apparent semicircle arcs, and the charge transfer resistance (*R*_ct_) of SrFe*_x_*Ni_1−*x*_O_3−δ_ (*x* = 0, 0.1, 0.2, 0.3, 0.4 and 0.5) can be derived from the diameter of the semicircle. The Z’-axis intercepts reflect the solution resistance (*R*_s_) basically fixed at 0.51 Ω cm^2^ and the oblique straight lines in low-frequency region represent the Warburg resistance (*Z*_w_) controlled by the electrode diffusion process. The Tafel curves of SrFe*_x_*Ni_1−_*_x_*O_3−δ_ perovskites are shown in Figure 14b, and the asymmetric curves reflect the irreversible redox reaction on the SrFe*_x_*Ni_1−_*_x_*O_3−δ_ perovskites. The *i*_0_ values of Tafel curves can be deduced from the intercepts when the overpotential (*η*) tends to zero, which relates to the electrocatalytic activity of SrFe*_x_*Ni_1−_*_x_*O_3−δ_ perovskites. In Table 5, the SrFe_0.3_Ni_0.7_O_2.85_ perovskite performs the attractive electrocatalytic activity (*i*_0_ = 891.3 × 10^−5^ mA cm^−2^) and conductivity (lower *R*_ct_ value of 7.58 Ω cm^2^) among the SrFe*_x_*Ni_1−_*_x_*O_3−δ_ perovskites, which agrees with the electrocatalytic properties (TN removal ratio and conductivity of ECR) in cleaning the nitrogenous wastewater.

## 4. Conclusions

In this work, low-cost SrFe*_x_*Ni_1−*x*_O_3−δ_ (*x* = 0, 0.1, 0.2, 0.3, 0.4 and 0.5) perovskites were fabricated using the citrate sol-gel method through doping Fe into the SrNiO_3_ matrix to improve the conductivity and electrocatalytic activity. In addition, the optimum conditions for fabricating SrFe*_x_*Ni_1−*x*_O_3−δ_ perovskites (reaction time of 120 min for citrate sol-gel, a calcination temperature of 700 °C and Fe doping content of *x* = 0.3) were successively obtained. Then SrFe*_x_*Ni_1−*x*_O_3−δ_ perovskites were coated on the Ti plate to prepare the SrFe*_x_*Ni_1−*x*_O_3−δ_/Ti electrode. The ECR was built with one SrFe*_x_*Ni_1−*x*_O_3−δ_/Ti anode and two stainless steel cathodes to clean nitrogenous wastewater. Furthermore, the characterization results strongly testify to the perovskite-type structure of SrFe*_x_*Ni_1−*x*_O_3−δ_. Finally, ECR with the SrFe_0.3_Ni_0.7_O_2.85_/Ti anode achieved the attractive TN removal ratio of 91.33% and conductivity of 3.62 mS cm^−1^ in the electrocatalytic process (electrocatalytic time of 150 min). In the optimum conditions, TN concentration in nitrogenous wastewater could be reduced below 15 mg L^−1^ and satisfied the discharge standard of pollutants for municipal wastewater treatment plants in China (GB 18918-2002, Class I-A Standard, TN ≤ 15 mg L^−1^). Therefore, the SrFe*_x_*Ni_1−*x*_O_3−δ_ perovskites have a significant and fascinating application for cleaning nitrogenous wastewater.

## Figures and Tables

**Figure 1:** Schematic diagram of the fabrication process of the SrFe*_x_*Ni_1−*x*_O_3−δ_ perovskites.

**Figure 2:** Schematic diagram of the preparation of the SrFe*_x_*Ni_1−*x*_O_3−δ_/Ti anode. (*N*,*N*-dimethylacetamide, DMAc; Polyvinylidene fluoride, PVDF)

**Figure 3:** Schematic diagram of the electrocatalytic reactor (ECR).

**Figure 4:** The effect of reaction time for citrate sol-gel on the electrocatalytic properties of SrFe*_x_*Ni_1−*x*_O_3−δ._

**Figure 5:** The effect of calcination temperature on the electrocatalytic properties of SrFe*_x_*Ni_1−*x*_O_3−δ._

**Figure 6:** The effect of Fe doping content (*x* value) in SrFe*_x_*Ni_1−*x*_O_3−δ_ on the electrocatalytic properties.

**Figure 7:** Characteristic parameters of SrFe*_x_*Ni_1−*x*_O_3−δ_ perovskites: Oxygen vacancy value (δ), tolerance factor (*t*), and 3d electron number in the B-site.

**Figure 8:** The effect of electrocatalytic time on TN concentration.

**Figure 9:** SEM images of (**a**,**b**) SrFe_0.3_Ni_0.7_O_2.85_ and (**c**,**d**) the surface of SrFe_0.3_Ni_0.7_O_2.85_/Ti anode.

**Figure 10:** FT-IR spectra of SrNiO_3_ perovskite and SrNiO_3_ precursor.

**Figure 11:** FT-IR (**a**) and Raman (**b**) spectra of SrFe*_x_*Ni_1−*x*_O_3−δ._

**Figure 12:** XRD patterns of SrFe*_x_*Ni_1−*x*_O_3−δ._

**Figure 13:** EDX spectrum of SrFe_0.3_Ni_0.7_O_2.85_ perovskite.

**Figure 14:** Electrochemical Impedance Spectroscopy (EIS) (**a**) and Tafel curves (**b**) of SrFe*_x_*Ni_1−*x*_O_3−δ._

**Table 1:** Components of materials for preparing the SrFe*_x_*Ni_1−*x*_O_3−δ_/Ti anode.

Anodic Materials	Mass Ratio (wt.%)	Function and Characteristic
SrFe*_x_*Ni_1−*x*_O_3−δ_ perovskites	56	Active material: stability, attractive electrochemical activity
Acetylene black	7	Conductor: huge specific surface area
Polyvinylidene fluoride (PVDF)	7	Binder: antioxidation, hydrophobicity
*N*,*N*-dimethylacetamide (DMAc)	30	Solvent: volatility, low toxicity

**Table 2:** The effect of different anodes in ECR for cleaning nitrogenous wastewater.

SrFe*_x_*Ni_1−*x*_O_3−δ_ Coated on the Anode	Voltage (V)	Power Density (mW cm^−2^)	Conductivity of ECR (mS cm^−1^)	TN Removal Ratio (%)
SrNiO_3_	6.97	82.0	3.38	37.21
SrFe_0.1_Ni_0.9_O_2.95_	6.68	78.6	3.52	49.75
SrFe_0.2_Ni_0.8_ O_2.9_	6.54	76.9	3.60	54.41
SrFe_0.3_Ni_0.7_O_2.85_	6.50	76.4	3.62	56.20
SrFe_0.4_Ni_0.6_O_2.8_	6.72	79.1	3.50	47.60
SrFe_0.5_Ni_0.5_O_2.75_	6.85	80.6	3.43	42.23

Total nitrogen (TN); Electrocatalytic Reactor (ECR).

**Table 3:** The optimum operation conditions and performance of ECR with the SrFe*_x_*Ni_1−*x*_O_3−δ_/Ti anode.

Item	Value
Anode	SrFe*_x_*Ni_1−*x*_O_3−δ_/Ti, 80.0 mm × 17.0 mm × 1.8 mm
Cathode	Stainless steel, 50.0 mm × 20.0 mm × 1.0 mm
Electrode gap	20.0 mm
Effective surface area of anode	5.10 cm^2^
Perovskite amount coated on the anode	0.09804 g cm^−2^
Electrocatalytic current identity	11.76 mA cm^−2^
Perovskite material for the anode of ECR	SrFe_0.3_Ni_0.7_O_2.85_
Reaction time for citrate sol-gel	120 min
Calcination temperature for SrFe*_x_*Ni_1−*x*_O_3−δ_	700 °C
Conductivity	3.62 mS cm^−1^
Initial TN concentration in wastewater	150 mg L^−1^
TN removal ratio	91.33%
Treatment time	150 min
Treatment volume	300 mL

**Table 4:** The relative content of elements in SrFe_0.3_Ni_0.7_O_2.85_ perovskite.

Elements	Weight Percent (%)	Atom Percent (%)
Sr	46.02	21.53
Ni	22.44	15.67
Fe	9.85	7.23
O	21.69	55.57
Total	100.00	100.00

**Table 5:** Parameters of SrFe*_x_*Ni_1−*x*_O_3−δ_ perovskites.

SrFe*_x_*Ni_1−*x*_O_3−δ_ Perovskites	*R*_ct_ (Ω cm^2^)	*i*_0_ (mA cm^−2^)
SrNiO_3_	17.88	2.570 × 10^−5^
SrFe_0.1_Ni_0.9_O_2.95_	11.54	54.95 × 10^−5^
SrFe_0.2_Ni_0.8_O_2.9_	9.97	158.5 × 10^−5^
SrFe_0.3_Ni_0.7_O_2.85_	7.58	891.3 × 10^−5^
SrFe_0.4_Ni_0.6_O_2.8_	13.85	37.15 × 10^−5^
SrFe_0.5_Ni_0.5_O_2.75_	15.88	12.02 × 10^−5^

## Supplementary Materials

The following are available online at http://www.mdpi.com/1996-1944/12/3/511/s1, Figure S1: Standard work curve of TN concentration, Figure S2: Effect of amount of SrFe*_x_*Ni_1−*x*_O_3−δ_ coated on the anode for the conductivity of ECR, Figure S3: Effect of amount of SrFe*_x_*Ni_1−*x*_O_3−δ_ coated on the anode for TN removal ratio, Table S1: UV Absorbances of various TN concentrations for standard work curve.
